# Evaluation of Antidiabetic and Antihyperlipidemic Activity of 80% Methanolic Extract of the Root of *Solanum incanum* Linnaeus (Solanaceae) in Mice

**DOI:** 10.1155/2022/4454881

**Published:** 2022-06-21

**Authors:** Yared Andargie, Woretaw Sisay, Mulugeta Molla, Getaye Tessema

**Affiliations:** School of Pharmacy, College of Medicine and Health Science, Debre Tabor University, Debre Tabor, Ethiopia

## Abstract

**Background:**

Conventional antidiabetic drugs are linked with a number of contraindications and untoward effects. The root decoction of *Solanum incanum* L. has traditionally been used to treat diabetes. However, its safety and efficacy have not been scientifically authenticated yet. Hence, the study was conducted in mice to corroborate its antidiabetic potential and safety profile.

**Methods:**

Using normoglycemic, oral glucose-loaded, and streptozotocin-induced diabetic mice models, the hypoglycemic and antihyperglycemic activities of 80% methanolic root extract were investigated. On streptozotocin-induced diabetic mice, the effect of the test extract on diabetic lipid profile and body weight was also investigated. Further, the in vitro *α*-amylase inhibition activity was assessed.

**Results:**

The test extract was safe at a limit test dose of 2 g/kg. Dose-dependent *α*-amylase inhibition activity was seen with peak percentage inhibition of 75.95% at 700 *μ*g/mL. In normoglycemic mice, the plant extract showed statistically significant hypoglycemic activity at 200 and 400 mg/kg (*P* < 0.001) at 6  h and 4 and 6 h of treatment, respectively; in oral glucose-loaded mice, at both the test doses, the glucose level was also significantly dropped at 120 (*P* < 0.01) and 60 and 120 min (*P* < 0.001), respectively; whereas, in the third model, the test extract showed significant antihyperglycemic activity at 100 mg/kg (*P* < 0.05) on the 14^th^ day and at 200 (*P* < 0.01) and 400 mg/kg (*P* < 0.001) on the 7^th^ and 14^th^ day of treatment. Similarly, following repeated administration of the test extract at 200 and 400 mg/kg, the body weight was significantly improved on the 14^th^ day (*P* < 0.05) and on the 7^th^ and 14^th^ day (*P* < 0.01), respectively, while diabetic dyslipidemia after 14 days (*P* < 0.05).

**Conclusion:**

The study revealed that the test extract showed promising antihyperglycemic and antihyperlipidemic activity. Thus, the findings back up its use in Ethiopian remedies for diabetes.

## 1. Background

Chronic hyperglycemia, hyperlipidemia, and hyperacidemia with reduced insulin secretion or action (or both) characterize diabetes mellitus (DM) [1]. The most frequent types of DM are type 1 and type 2, with type 1 caused by the inability of the body to produce adequate insulin, whereas type II diabetes mellitus is characterized by fasting hyperglycemia due to insulin resistance [2].

Currently, diabetes is becoming a major concern globally and a leading cause of morbidity and mortality in most countries, with an estimated 382 million adults exposed and 5.1 million people died in 2013 [2]. According to World Health Organization (WHO) data, the number of diabetics has grown from 108 million in 1980 to 422 million in 2014 [3]. It is predicted that 592 million people will be affected by the disease in 2035, with the greatest increase in low- and middle-income countries [4]. Ethiopia is one of the top five countries in Sub-Saharan Africa with the highest number of people affected by diabetes mellitus [3].

The use of medicinal plants has been a part of human endeavors to combat diseases for millennia, including diabetes mellitus. The World Health Organization estimated that approximately 80 percent of the population in developing countries relies on herbal products, which are considered to be affordable, easily available, and less toxic [5, 6]. Currently, nearly 25% of drugs in modern pharmacopeia are descended from natural products that were first used in traditional medicine. Taking metformin as an example, it was originally isolated from the medicinal plant *Galega officinalis* and is now prescribed in modern medicine to treat diabetes [7].

An ethnobotanical survey revealed that a diverse range of medicinal plants are being used to treat the disease in many ethnic societies around the world, with *S. incanum* L. being one of these plants in Ethiopian folkloric medicine [8]. Among these, a number of medicinal plants, including *Allium sativum*, *Aloe vera*, *Coccinia indica*, *Eugenia jambolana*, *Falcaria vulgaris*, *Calpurnia aurea*, *Hagenia abyssinica*, and *Stevia rebaudiana*, have been thoroughly studied for their antidiabetic efficacy [9–11]. To date, however, there has been no scientific validation of the therapeutic potential and safety profile of the root of *Solanum incanum* L.

*Solanum incanum* L., also known as Sodom or bitter apple (in English), is a member of the Solanaceae family that grows in many parts of Africa, the Middle East, and Far East Asia. It is a perennial shrub-like herb with small prickles on the leaves and stems that can grow up to 1.8 meters. When ripe, the fruits are small berries that measure 2–3 cm in diameter and are yellowish orange or brown in color [12, 13]. It is a very common shrub in Ethiopia, where it can be found on abandoned agricultural lands, along roadsides, and in village yards. The plant has several local names in Ethiopia: Embuay (in Amharic) and Hiddii (in Oromifa) [13].

Traditionally, various parts of the plant have been used to treat a number of diseases. Aliments like angina, stomachaches, colic, headaches, and fever are relieved with the root segment of the plant. Other medicinal uses include relieving pain in patients with menstruation, liver disease, onchocerciasis, pleurisy, pneumonia, and rheumatism [14]. Other plant parts are also commonly used to treat a wide range of dermatological problems, including ringworm, burns, sores, rashes, wounds, warts, carbuncles, inflammations, and benign tumors [15]. In the Libo Kemkem district, in the Amhara region of Ethiopia, it is claimed that the root part chewed and then taken as a juice has been used to treat diabetes mellitus [8].

There have been numerous experimental studies that proved various parts of the plant have a variety of activities, including *in vitro* antimicrobial activity of the leaf, fruit, and stem extract [16]; analgesic and spasmolytic activity of the leaf extract [17]; anti-inflammatory and antinociceptive effects of the root extract [14]; antihyperlipidemic effect of the fruit extract [18]; *in vitro* antiprotozoal activity of the leaf extract [19]; wound healing and anti-inflammatory activity of the leaf extract [15]; and antischistosomal activity of the root extract [20].

Despite the fact that a variety of medications are available for treating DM, they have been linked to a number of unintended side effects. Thus, it has been suggested to use natural products as effective pharmaceutical alternatives [21]. The root of *S. incanum* L. has been used to treat diabetes in Ethiopian folklore medicine without any scientific evidence to support its safety and efficacy. Hence, the current study sought to validate the *in vitro* and *in vivo* antidiabetic activity of an 80% methanolic extract of the root of *S. incanum* L. Additionally, the study aimed to provide a clue about the nature of the bioactive principles of the plant that are responsible for its action.

## 2. Materials and Methods

### 2.1. Drugs, Chemicals, and Instruments

The drugs, chemical reagents, and instruments used in the experiment were absolute methanol 99.9% (Nice Chemicals, India), streptozotocin (Fisco Research Laboratories), glibenclamide 5 mg (Julphar Pharmaceuticals, Ras Al Khaimah, UAE), acarbose 50 mg (Bayer), porcine pancreatic *α*-amylase (Molychem), citric acid monohydrate 99% (Lab Tech Chemicals, Mumbai, India), 50 mM trisodium citrate dihydrate (Blulux Laboratories, Faridabad, India), 40% glucose solution (Reyoung Pharmaceuticals, Shandong, China), blood glucose meter and strips (Alliance International, Taiwan), clinical chemistry analyzer (Shenzhen Mindray Bio-Medical Electronics Co., Ltd, China), Wagner's reagent (Research-Lab Fine Chem Industries, India), lead acetate 1% (Guangdong Guanghua Chemicals Factory, China), sodium hydroxide 48% (BDH, chemical lab, England), ferric chloride 12% and sulfuric acid 98% (BDH Laboratory Supplies Poole, England), chloroform (Hi-Media Laboratory Reagents, India), UV-visible spectrophotometer (Agilent Technologies), and lyophilizer (Labfreez Instruments Group Co., Ltd., Japan). All supplies were of analytical grade and obtained from governmental and private suppliers.

### 2.2. Experimental Animals

Healthy male Swiss albino mice (25–30 g) purchased from the Ethiopian Public Health Institute, Addis Ababa, were used to undergo the study. Except for the oral toxicity investigation, female mice were excluded due to males' high compatibility with the models [22]. The animals were kept in a conducive environment in plastic cages with softwood shavings as bedding and free access to pellet food and water. They were acclimatized to the laboratory environment for one week before starting the main experiment. Throughout the experiment, animals were handled and cared for in accordance with international laboratory animal use and care guidelines, and the study was accepted by the Research and Ethics Committee of College of Medicine and Health Science, Debre Tabor University, with reference number SOP 1/106/14.

### 2.3. Plant Material Collection and Preparation

In January 2021, fresh *Solanum incanum* L. roots were collected in the Libo Kemkem district, South Gondar zone, Amhara region, Northwest Ethiopia. Following collection, a botanist performed taxonomic verification, and the plant specimen was stored in the botanic garden of the Department of Biology, University of Gondar, with the registration number AY01 for future reference. The roots of the plant were then harvested in bulk, gently cleaned with tap water, and air dried for two weeks at a standard temperature. The roots were then grounded into a coarse powder and stored in a plastic container until they were needed for extraction.

### 2.4. Preparation of the Crude Extract

The crude extract of the root of the plant was obtained using the following procedure with minor modifications [23]. A total of 600 g of coarsely powdered plant root was macerated in 80% methanol for 72 h with intermittent hand shaking. The extract was separated from the marc with gauze after 72 h and then filtered through Whatman filter paper No. 1. The residue was then re-macerated twice for more three days, for a total of six days, with a fresh solvent of 80% methanol to exhaustively extract the plant material. To remove methanol, the marc was pressed, and the filtrates from each extraction were mixed and evaporated in a hot oven set at 40°C. The extract was further condensed to dryness by freeze-drying using a lyophilizer. Finally, the crude extract percentage yield was computed and maintained in an airtight container in the refrigerator at 4°C until employed for the intended experiment.

### 2.5. Qualitative Phytochemical Screening Test

The crude extract of the root of *Solanum incanum* L. was screened for the presence of active secondary metabolites by using standard assays [24]. Thus, assays for alkaloids, saponins, flavonoids, terpenoids, phenols, steroids, glycosides, tannins, and anthraquinones were implemented in the study.

### 2.6. Quantitative Determination of Phytochemicals

#### 2.6.1. Determination of Flavonoid Content

Estimation of flavonoid content in the test extract was performed by using the following procedure [25]. In a 250 mL beaker, 2.50 g of sample was added to exactly 50 mL of 80% methanol, covered, and left to stand at 25°C for 24 h. Just after disposing of the supernatant, the remnant was re-extracted three times with the same amount of ethanol. For filtration, Whatman filter paper No. 42 (125 mm) was used. After that, each sample filtrate was poured into a beaker and dried using a water bath. Then, using a desiccator, the dried filtrate was cooled and weighed till a steady weight was attained. Eventually, the content of flavonoids was estimated in percentage by using the algorithm below:

(1) $$\begin{array}{c} \text{Flavonoid content}\left(\%\right)=\frac{\text{Weight of flavonoid}}{\text{Weight of sample}}\times 100. \end{array}$$

#### 2.6.2. Determination of Phenolic Content

By employing a Folin–Ciocalteu's reagent microplate assay technique, the phenolic content of the test extract was estimated using the previous method with minor modifications. Using a standard graph constructed with gallic acid, the quantity of the phenols in the extract was measured and expressed as gallic acid equivalent per gram of extract [26].

#### 2.6.3. Determination of Alkaloid Content

The content of alkaloids was determined by using the following method as explained by Ezeonu and Ejikeme [25]. In a 250 mL beaker, 2.50 g of powdered sample was poured into ethanol with 200 mL of 10% acetic acid and left to stand for 4 h. In a water bath, soon after filtration, the extract was concentrated to one-quarter of its baseline volume. Then, 15 drops of concentrated ammonium hydroxide was slowly added to the extract until complete precipitation was observed. Following 3 h of precipitation, the filtered liquid was disposed of and the residuals were carefully rinsed with 20 mL of 0.1 M ammonium hydroxide. Afterward, using Gem filter paper (12.5 cm), the mixture was filtered. Then, the residue was concentrated in a hot oven set at 40°C, and the weight was measured by using an electronic balance. Finally, using this formula, the quantity of alkaloid was estimated and expressed in percentages:

(2) $$\begin{array}{c} \text{Alkaloid content}\left(\%\right)=\frac{\text{Weight of alkaloid}}{\text{Weight of sample}}\times 100. \end{array}$$

### 2.7. Investigating In Vitro *α*-Amylase Inhibitory Effect

The *α*-amylase inhibition assays were conducted through 3,5-dinitrosalicylic acid (DNSA) technique with minor modifications [27]. The sample extract of *S. incanum* L. was diluted in buffer (Na_2_HPO4/NaH_2_PO4 (0.02 M), NaCl (0.006 M) at pH 6.9) to obtain concentrations ranging from 100 to 700 *μ*g/mL. 200 *μ*L of porcine pancreatic *α*-amylase solution (2 units/mL) was blended with the same volume of the plant extract and was incubated at 30°C for 10 min. After that, each tube was filled with 200 *μ*L of starch solution (1% in water (w/v)) and incubated for 3 min. The reaction was stopped by adding 200 *μ*L of DNSA reagent (12 g of sodium potassium tartrate tetrahydrate in 8.0 mL of 2 M NaOH and 20 mL of 96 mM of 3,5-dinitrosalicylic acid solution) to a water bath at 90°C and boiling for 10 min. After the solution was cooled down at room temperature, the absorbance was then measured at 540 nm using a UV-visible spectrophotometer and diluted with 5 mL of distilled water. The blank with 100% enzyme activity was produced by substituting the sample extract with 200 *μ*L of the buffer. A positive control sample was made with acarbose, and the reaction was carried out in the same way as the plant extract reaction. The inhibition of *α*-amylase was computed using the formula below and expressed as a percentage of inhibition; and the IC_50_ values were calculated by plotting the percent *α*-amylase inhibition versus sample extract concentration:

(3) $$\begin{array}{c} \%\text{inhibition}=\frac{\text{Abs control}-\text{Abs sample}}{\text{Abs control}}\times 100, \end{array}$$

where Abs control = absorbance of control and Abs sample = absorbance sample.

### 2.8. Acute Toxicity Study

Acute oral toxicity of the crude extract was tested on healthy, nonpregnant, and adult female Swiss albino mice according to the OECD-425 guideline. As a result, five 6- to 8-week-old female albino mice were employed. All animals were starved for 3 h before and 2 h after receiving the test extract. For the first animal, a limit test dose of 2 g/kg was given. The mouse was then closely monitored for the next 4 h, every 30 min, for any signs of toxicity or mortality within the first 24 h. Based on the results of the first animal, four more mice were given a similar dose of the test extract in a sequential order. The animals were then monitored for 14 days for any signs of overt toxicity or mortality [28].

### 2.9. Grouping and Dosing of Animals

Because male mice were more susceptible to streptozotocin (STZ) than females, they were employed in all animal models (normoglycemic mice, oral glucose-loaded mice, and repeated dose treated diabetic mice) [29].

The animals were randomly allocated into five groups in the normoglycemic and oral glucose-loaded mice models, each having six mice. In both models, Group I (negative control) received 10 mL/kg distilled water (DW), while Group II, III, and IV were given 100, 200, and 400 mg/kg test extract, respectively. Meanwhile, Group V (positive control) was given the reference drug (glibenclamide 5 mg/kg). In both the models, a single dose of the respective treatments was given.

In an STZ-induced diabetic experiment, mice were randomly allocated into six groups (5 groups of diabetic mice and one group of normal mice), each having six mice. Group I (negative control) and Group VI (normal control) were given 10 mL/kg DW. Group II, III, and IV (tested groups) received 100, 200, and 400 mg/kg of the test extract, respectively, while Group V (positive control) was treated with 5 mg/kg GLC. In this model, the treatments were given for 14 days.

Based on previous research findings, glibenclamide (5 mg/kg) was chosen as the standard medication [30]. The doses of the test extract to be given were calculated by using the acute toxicity study results, and the volume of administration was 1 mL/100 g of body weight of the mouse [28]. *Solanum incanum* L. is historically used by the community through the oral route for treating DM. Thus, the study was carried out by utilizing this method of administration [8].

### 2.10. Measurement of Blood Glucose Level

In all animal models, blood samples were taken from the tail vein of each starved mouse by cutting the tip of the tail aseptically, and blood glucose levels (BGLs) were determined by using a blood glucose meter with a test strip. Blood glucose measurements were made three times in all models, and the average value was taken.

### 2.11. Induction of Experimental Diabetes

Streptozotocin (STZ) was used to induce diabetes in this study and was initially dissolved in 0.1 M cold citrate buffer (pH = 4.5) before being used. Then, after starving the animals for 16 h, the freshly produced STZ solution at 150 mg/kg was administered intraperitoneally [31]. Following 30 min of receiving STZ injection, the animals were given food and water. To avoid death due to hypoglycemic shock, the animals were given 5% glucose solution for 24 h after 6 h of receiving STZ. Three days after being given STZ, mice having fasting blood glucose levels greater than 200 mg/dl were included in the trial as diabetic [32]. Soon after being screened, STZ-induced diabetic animals were allocated randomly into separate groups to carry out the experiment.

#### 2.11.1. Assessing the Hypoglycemic Activity of the Crude Extract in Normoglycemic Mice

Normal mice were randomly assigned into five different groups, each having six after being fasted overnight. The animals were then given DW, plant extract, and the reference drug according to their groups as specified in Section 2.9. Thereafter, the BGL was measured in each mouse immediately before treatment (at 0 h) as a baseline and then at 1, 2, 4, and 6 h of treatment [33].

#### 2.11.2. Assessing the Glucose-Lowering Effect of the Crude Extract on Oral Glucose-Loaded Mice

After starving overnight for 14 h, mice were randomly allocated into 5 groups, each having six, and treated as stated under Section 2.9. Then, the baseline blood glucose level was measured. After 30 min of extract administration, each mouse was given 2 g/kg of glucose solution orally. The BGL of each mouse was measured just before treatment (at 0 min) as a baseline and then at 0.5, 1, and 2 h of glucose administration [34].

#### 2.11.3. Evaluating the Effect of Repeated Dose of the Crude Extract on Antihyperglycemic Activity and Body Weight in STZ-Induced Diabetic Mice

In the repeated dose STZ-induced diabetic model, the mice were placed into six groups, each having six. The vehicle, reference medication, and test extract were given once daily for 14 days as indicated in Section 2.9. Following a 14-h overnight fasting, the BGL and body weight of mice were recorded just before treatment (day 0) and on the 7^th^ and 14^th^ day of treatment [35].

#### 2.11.4. Evaluating the Effect of the Test Extract on Serum Lipid Level of STZ-Induced Diabetic Mice

Overnight fasting mice were killed on the 15^th^ day of treatment with an overdose of pentobarbitone (150 mg/kg, ip), and blood samples were obtained in a sterile tube through cardiac puncture [36]. After 2 h of storing at a standard temperature, the blood samples were centrifuged at 30°C for 15 min at 2500 rpm. Using an automated chemistry analyzer, the supernatant was then separated from the precipitate and serum samples were prepared to determine the levels of triglyceride, TC, HDL, LDL, and VLDL cholesterol [37].

### 2.12. Statistical Analysis

The data were entered and processed using SPSS software, version 24 [38]. The experimental data were expressed as mean ± standard error of the mean (SEM), and statistical significance was determined by using one-way analysis of variance (ANOVA) followed by Tukey's post hoc test for multiple comparison. When the *P*-value was less than 0.05, the results were considered statistically significant.

## 3. Results

### 3.1. Extraction Yield of Plant Material

At the end of maceration, 99 g of dried yellowish brown semisolid extract (percentage yield, 16.5% w/w) was obtained.

### 3.2. Phytochemical Screening Test

As per preliminary phytochemical testing, bioactive constituents such as flavonoids, alkaloids, phenols, tannins, saponins, terpenoids, steroids, and anthraquinones were detected in the hydro-methanolic extract of the root of *S. incanum* L. (Table 1).

### 3.3. Quantitative Determination of Phytochemicals

The amounts of total flavonoids, phenolics, and alkaloids determined in the test extract are presented as shown in Table 2. The content of flavonoids in the sample test extract was 0.21 g (8.4%), while the phenolic content was 74.51 mg/g (7.5%). Besides, the alkaloid content was quantified and has been found to be 0.03 g (1.2%).

### 3.4. Acute Oral Toxicity Study

During the 14-day follow-up period, there was no mortality after a single dose administration of 2 g/kg of the test extract. As a result, the test extract's median lethal dose (LD_50_) is predicted to be greater than 2 g/kg. Furthermore, there were no signs or symptoms of toxicity in the study, such as behavioral, neurological, autonomic, or somatic abnormalities.

### 3.5. In Vitro *α*-Amylase Inhibitory Effect

The percent *α*-amylase inhibition activity is plotted as a function of sample extract and acarbose concentration as shown in the graph below (Figure 1). For varied concentrations of the sample extract and the reference drug, concentration-dependent inhibition was observed. The crude root extract of *S. incanum* L. showed maximal *α*-amylase enzyme inhibition activity of 75.95% at 700 *μ*g/mL, with an IC_50_ of 495 *μ*g/mL. Correspondingly, the peak percentage inhibition (89.69%) was seen with the standard drug (acarbose) at a similar concentration, with an IC_50_ of 393 *μ*g/mL.

There was no statistically significant difference between the IC_50_ of acarbose and the sample extract (*P* > 0.05).

### 3.6. Effects of the Crude Extract on the Normoglycemic Mice Model

The effect of the test extract on fasting BGL in nondiabetic mice at various time points when compared with negative control is shown in Table 3. There was no statistically significant variation in baseline blood glucose levels among the groups. At 1- and 2-h time points, none of the tested groups showed a statistically significant reduction in blood glucose levels. Similarly, groups given the standard drug did not also reduce blood glucose levels significantly at 1 h of treatment. However, a significant drop in the BGL was observed in groups given 200 mg/kg at 6 h (*P* < 0.001) and 400 mg/kg of the test extract at 4- and 6-h (*P* < 0.001) time points. However, at all time points, a reduction in the BGL at 100 mg/kg was negligible (*P* > 0.05). In addition, when comparing the standard drug with the vehicle, the standard drug's effect was evaluated and found to be statistically significant at 2, 4, and 6 h of treatment (*P* < 0.001). When the standard medicine-treated groups were compared with 100 mg/kg treated groups, the drop in the fasting BGL was statistically significant at 4- and 6-h time points (*P* < 0.001); whereas the drop was statistically significant (*P* < 0.01) at 6 h of treatment when compared with 400 mg/kg treated group.

### 3.7. Effects of the Crude Extract on Oral Glucose-Loaded Mice Model

The effect of *S. incanum* L. crude extract on oral glucose-loaded nondiabetic mice is summarized in Table 4. Before the animals were treated with their respective treatments, there was no significant difference in fasting BGLs across the groups. Thirty minutes after oral administration of 2 g/kg glucose to normal mice, the peak BGL was observed in each group (Figure 2). It is intended to mean that the test extract showed significant reduction in hyperglycemia at 400 mg/kg at 60 and 120 time points (p<0.001). Correspondingly, when compared with the negative control, groups given GLC showed a substantial improvement in hyperglycemia (*P* < 0.001) at the aforementioned time points. Nonetheless, the crude extract at the lowest dose (100 mg/kg) was unable to elicit detectable changes at all time points. When compared with the 100 and 200 mg/kg test extract-treated groups, the standard drug (GLC) substantially reduced hyperglycemia at 1- and 2-h (*P* < 0.001) time points, and similarly at 1 (*P* < 0.01) and 2 h of treatment (*P* < 0.05) when compared with groups given 400 mg/kg of the test extract.

### 3.8. Effects of Repeated Daily Doses of the Crude Extract in STZ-Induced Diabetic Mice

After inducing the animals with STZ, the fasting BGL was measured once weekly in both normal and diabetic mice treated with the test extract, distilled water, and the standard drug. The findings are presented in Table 5. In diabetic mice, compared with the normal control group, a marked and statistically significant rise in the fasting BGL was seen after induction (*P* < 0.001). In all groups of diabetic mice, however, there was no significant variation in the baseline fasting BGL. When compared with the diabetic control, those groups given the test extract at 100 mg/kg (*P* < 0.05, on the 14^th^ day), 200 mg/kg (*P* < 0.01, on the 7^th^ and 14^th^ day), and 400 mg/kg (*P* < 0.001) at both time points had significantly lower blood glucose levels. Likewise, groups receiving the standard drug experienced a significant (*P* < 0.001) decrease in the BGL on the 7^th^ and 14^th^ day. The test extract at 100 mg/kg, on the other hand, failed to show a drop in blood glucose on the 7^th^ day when compared with the diabetic control. Similarly, neither GLC nor *S. incanum* L. treatment was able to restore normal blood glucose levels in diabetic mice as in the normal control mice.

### 3.9. Effects of Repeated Daily Doses of the Crude Extract on the Body Weight of STZ-Induced Diabetic Mice

The effect of repeated daily doses of the extract on body weight of diabetic mice is presented in Table 6. Before STZ induction, there was no statistically significant variation in the body weight of mice among all groups. The weight of mice was recorded as a baseline after 3 days of induction, and there was no significant difference between the diabetic groups (*P* > 0.05). However, when compared with the normal control, there was a substantial weight loss (*P* < 0.01). As compared with normal mice, STZ-induced diabetic mice showed considerable body weight loss on the 7^th^ and 14^th^ day. The findings demonstrated that the test extract at 200 (*P* < 0.05, on the 7^th^ day) and 400 mg/kg (*P* < 0.01, on the 7^th^ and 14^th^ day) doses exhibited significant improvement in body weight relative to the diabetic control. However, it was still less than that in the normal control group. Similarly, the body weight of diabetic groups received the reference drug were also increased dramatically (*P* < 0.001). In comparison with the normal control, however, the body weight of the diabetic control was drastically declined (*P* < 0.001) on both days.

### 3.10. Effects of Repeated Daily Doses of the Crude Extract on Serum Lipid Levels of Diabetic Mice

As compared with normal control, there was a notable (*P* < 0.001) increase in the serum levels of TC, TG, LDL, and VLDL cholesterol after the induction of diabetes, but a significant reduction (*P* < 0.001) in HDL cholesterol (Table 7). At a lower dose (100 mg/kg), the test extract had no significant impact on the serum levels of all the aforementioned indices relative to diabetic control. The test extract at 200 mg/kg, on the other hand, resulted in a significant reduction in serum levels of TG (*P* < 0.01) and TC and LDL-c (*P* < 0.05). However, the effect on VLDL-c and HDL-c levels in the serum was found to be negligible. Furthermore, the effect of the test extract at 400 mg/kg was assessed and dramatically lowered the serum levels of TC (*P* < 0.01), TG (*P* < 0.001), and LDL-c (*P* < 0.01), while raising the serum level of HDL-c (*P* < 0.05) as compared with the diabetic control. Correspondingly, the standard drug GLC also significantly halved the serum levels of TC, TG, LDL-c, and VLDL-c, while boosting HDL cholesterol. However, the standard drug and the test extract were unable to normalize the serum level of all parameters as in the normal control mice.

## 4. Discussion

Human beings frequently utilize various segments of medicinal plants as a treatment for a variety of diseases, including diabetes, despite the lack of scientific evidence supporting their safety and efficacy [4]. As a result, it is critical to adequately assess the safety and efficacy profile of medicinal herbs utilized in traditional medicine. As conventional antidiabetic drugs have limitations, the need for novel, more efficient, less-expensive, and nontoxic medications has become a top priority. Thus, the search for alternative therapies derived from natural products is highly demanding as they are thought to be safe and easy to obtain and do not require time-consuming pharmaceutical production [39].

In an acute oral toxicity study, during the 14-day follow-up period, administration of the crude test extract at a single limit test dose of 2 g/kg did not cause mortality or delayed toxicity. The findings demonstrated that the test extract's LD_50_ value is expected to be more than 2 g/kg, showing a large margin of safety. Overall, the results showed that the root of the plant extract is palatable and nontoxic, indicating that the plant can be used safely in traditional settings.

In this study, before commencing an *in vivo trial*, the antidiabetic effect of *S. incanum* L. root extract was examined *in vitro* by measuring the *α*-amylase inhibitory activity. Inhibition of starch-metabolizing enzymes such as *α*-amylase is the current treatment strategy for managing diabetes and its consequences since the enzyme controls the catabolism of starch into glucose [40]. The findings on *S. incanum* L. root extract showed concentration-dependent inhibition of *α*-amylase activity. The IC_50_ value of the plant extract is 495 *μ*g/mL, while the IC_50_ value is 393 *μ*g/mL for the standard drug “acarbose,” a widely used antidiabetic drug.

The results revealed that the plant extract may have antidiabetic properties. Polyphenolic metabolites such as flavonoids, tannins, and phenolic acids have inhibitory activity against the aforementioned enzyme [21]. In this study, the phytochemical analysis revealed that the extracts are enriched in polyphenolic compounds. Hence, the extract's *α*-amylase inhibitory effect could be attributed to the presence of such secondary metabolites.

Numerous phytochemical components extracted from various plant species are thought to have significant hypoglycemic, antihyperglycemic, and glucose-lowering capabilities. Some of the bioactive components are flavonoids, triterpenoids, alkaloids, and phenolics [6]. The aforementioned activity could be accomplished by augmenting insulin release from pancreatic *β*-cells, diminishing glucose absorption in the small intestine, increasing glucose consumption in the body, and/or initiating glycogenesis in the liver [41]. In addition, these active phytochemical compounds have been scientifically proven to regenerate damaged beta-cells while shielding them from oxidative stress in diabetic rats [42].

Streptozotocin-induced diabetes in mice is the most extensively used and standardized model of experimental diabetes. Usually, it is favored to use this diabetogenic agent over alloxan because of its repeatability and wider species effectiveness. Literature indicates that the inducer at a single dose (150 mg/kg) can cause sustained hyperglycemia in mice for at least one month [30]. Similarly, at this dose, the chemical causes chronic hyperglycemia with no substantial fluctuation in blood glucose levels for two weeks, as shown in the diabetic control.

According to a phytochemical assay, secondary metabolites such as saponins, tannins, terpenoids, phenols, flavonoids, glycosides, steroids, and anthraquinones were found in the crude extract of *S. incanum* L. Hence, the diverse bioactive phytochemical components detected in hydro-methanolic extracts of the root of the plant may be responsible for the observed glucose-lowering and antihyperglycemic effect.

The *in vitro* finding established the candidacy for further analysis of the antidiabetic activity of the test extract in *in vivo* models. The effect of the extract on BGLs was evaluated by initiating normoglycemic, oral glucose-loaded, and STZ-induced diabetic mice models. In the normoglycemic mice model, the vehicle-treated group did not exhibit a statistically significant drop in fasting blood glucose levels. Nondiabetic mice, however, showed a substantial reduction in blood glucose levels after being given 200 mg/kg (*P* < 0.001) test extract at 6-h time point and 400 mg/kg (*P* < 0.001) test extract at 4- and 6-h time points. The hydro-methanolic extract's hypoglycemic effect was found to be time-dependent, with the peak effect occurring at 4 and 6 h of treatment. This suggested that the bioactive elements in the plant extract required more time to achieve a sufficient concentration at the target site.

The standard medicine has been shown to have antidiabetic action, possibly through enhancing insulin release from pancreatic *β*-cells and inhibiting glucagon secretion [43]. Flavonoids and tannins obtained from natural products have been shown to induce insulin release from pancreatic *β*-cells [44]. Since these secondary metabolites exist in *S. incanum* L. root extract, the test extract's hypoglycemic activity could be attributed to a mechanism similar to that of glibenclamide.

The OGTT is a test to assess the body's ability to use glucose and is the “gold standard” for diagnosing diabetes mellitus [45]. In this experiment, the findings revealed that administration of *Solanum incanum* L. root extract showed a significant dose-dependent reduction of BGL in oral glucose-loaded mice. Following glucose administration, the test extract at 200 mg/kg showed a statistically significant reduction in the BGL at 60 (*P* < 0.05) and 120 min (*P* < 0.01). However, at both time points, the effect of the test extract at the higher dose (400 mg/kg) was extremely significant (*P* < 0.001), indicating that the crude extract had reached its peak antihyperglycemic action at the highest dose. This could be owing to the test extract's sufficient concentration of active phytochemicals at this dose.

The antihyperglycemic potential of the test extract could be attributed to suppression of glucose absorption, enhancement of peripheral glucose consumption, reduction in glycogenolysis, and gluconeogenesis [46]. Blocking glucose absorption by inhibiting intestinal *α*-glucosidase and pancreatic *α*-amylase activity has been shown in studies to reduce postprandial hyperglycemia [47]. Thus, the test extracts' glucose-lowering effect could be associated with its *α*-amylase inhibitory activity as confirmed by the *in vitro* study.

In STZ-induced diabetic mice, the highest reduction in the blood glucose level was observed on the 14^th^ day at 400 mg/kg of the crude extract. The percentage reduction (19.7%) was comparable to the standard drug (33.7%). It was observed that the test extract activity was found to be dose dependent. This could signify that the bioactive chemicals of the plant which are crucial for antidiabetic activities are more concentrated at higher doses. Therefore, the current investigation speculated that the hydro-methanolic extracts of the root of *S. incanum* L. have remarkable antidiabetic activity on STZ-induced diabetic mice in a time- and dose-dependent manner.

The findings suggested that the test extract may have a potent antihyperglycemic effect. There are plausible reasons related to this finding. It has been proposed that the use of antioxidants can help prevent diabetic complications by reducing oxidative stress [48]. The primary causes of the etiology and progression of diabetes are oxidative stress and inflammation [49]. Streptozotocin causes diabetes mellitus by preferentially destroying the pancreatic beta-cells. Studies have shown that when given to rodents, it induces the death of *β-*cells after three days [4]. Findings reported that *S. incanum* L. root extract had significant *in vitro* antioxidant activity [23]. This implied that the antihyperglycemic activity in STZ-induced diabetic mice could be owing to its *β*-cell protecting effect against oxidative free radicals.

The mechanism of action of the plant extract could have been due to the release of insulin from pancreatic beta-cells. The existence of diverse bioactive principles that have been implicated in hypoglycemic activity might explain the antidiabetic effect of the hydro-methanolic root extract of *Solanum incanum* L. [50]. Flavonoids, sterols, and saponins have been found in ethanoic fruit extracts of *L. camara* L., which have been shown to have hypoglycemic effects in STZ-induced diabetic rats [51].

When STZ-induced diabetic mice were compared with normal mice, they lost a significant amount of body weight (*P* < 0.01). The weight loss in diabetic mice might be linked to insulin insufficiency, which causes tissue protein breakdown and fat catabolism in adipose tissues [52]. However, the body weight of mice was significantly increased at 200 and 400 mg/kg of plant extract. The capability of the test extract to improve body weight may be attributable to the presence of bioactive chemicals that suppress free radical formation through hyperglycemia. It might also be done by preventing muscle atrophy caused by poor glycemic control, which leads to body weight loss [53].

Hypertriglyceridemia and hypercholesterolemia are the most frequent lipid abnormalities in diabetes. It is characterized by high serum TG, TC, LDL-C, and low HDL-C levels. Insulin shortage activates hormone-sensitive lipase, resulting in increased lipolysis and VLDL synthesis from the liver. Also, during insulin deficiency, the activity of lipoprotein lipase is reduced that could lead to a decreased clearance of chylomicrons and VLDL [30]. Repeated administration of *Solanum incanum* L. root extract for 14 days significantly reduced STC, STG, VLDL-c, and LDL-c levels while increasing HDL-c levels in a dose-dependent manner. This finding was in consonance with other findings that proved the aqueous ethanol and n-butanol fraction of *M. stenopetala* leaves had notable antihyperglycemic and dyslipidemic activity [4]. Reduced cholesterogenesis and fatty acid production by inhibition of pancreatic cholesterol esterase and pancreatic lipase, respectively, may possibly explain the reported antihyperlipidemic effect [54, 55].

## 5. Conclusions

These findings confirmed that the crude extract of *S. incanum* L. root possesses antihyperglycemic and antihyperlipidemic activity. The presence of diverse bioactive phytochemicals such as flavonoids, tannins, terpenoids, phenols, saponins, phenols, alkaloids, and anthraquinones may be implicated in the aforementioned activities. Based on the findings of the study, it is plausible to conclude that the root of *S. incanum* L. can be utilized as an alternative supplement in Ethiopian folkloric medicine to treat diabetes. Further investigation is required to explore how the plant extract modulates blood glucose and lipid levels.

## Figures and Tables

**Figure 1:** *α*-Amylase inhibition (%) as a function of *Solanum incanum* L. extract and acarbose concentration.

**Figure 2:** Effect of *S. incanum* L. crude extract on the blood glucose level of oral glucose-loaded mice.

**Table 1:** Preliminary phytochemical screening of hydro-methanolic extract of *S. incanum* L. root extract.

Phytochemical constituents	Methods used for screening	Result
Flavonoids	Lead acetate test	Positive
Terpenoids	Salkowski's test	Positive
Alkaloids	Wagner's test	Positive
Phenols	NaOH test	Positive
Tannins	Ferric chloride test	Positive
Saponins	Foam test	Positive
Steroids	Salkowski's test	Positive
Glycosides	Glycoside test	Negative
Anthraquinones	Borntrager's test	Positive

Positive: present, Negative: absent.

**Table 2:** Total flavonoid, phenolic, and alkaloid contents of *Solanum incanum* L. root extract.

Test extract	Flavonoid content (g)	Phenolic content (mg/g)	Alkaloid content (g)
*Solanum incanum* L.	0.21 (8.4%)	74.51 (7.5%)	0.03 (1.2%)

**Table 3:** Hypoglycemic activity of hydro-methanolic root extract of *Solanum incanum* L. in normoglycemic mice.

Group	Blood glucose level (mg/dl)				
	Baseline	1 h	2 h	4 h	6 h
DW10	123.70 ± 1.18	121.88 ± 1.37	122.43 ± 0.86	123.43 ± 0.69^d3^	122.77 ± 1.00^c3d3^
SIRE100	124.53 ± 1.10	122.04 ± 0.91	123.65 ± 0.80	123.66 ± 0.85^d3^	122.80 ± 0.78^c3d3^
SIRE200	125.12 ± 0.74	123.99 ± 0.88	123.32 ± 0.66	123.64 ± 0.66^d3^	112.16 ± 0.86^a3b3d1^
SIRE 400	124.70 ± 0.65	123.50 ± 0.72	123.40 ± 0.60	112.28 ± 1.04^a3b3c3^	108.24 ± 0.60^a3b3c1^
GLC5	124.66 ± 0.64	119.99 ± 0.78	108.40 ± 1.00^a3b2c2d1^	100.16 ± 0.99^a3b3c3d1^	95.05 ± 0.87^a3b3c3d2^

Results are expressed as mean ± SEM (*n* = 6) and analyzed by one-way ANOVA followed by Tukey's post hoc test. ^a^ Compared with the negative control,^b^ compared with SIRE 100 mg/kg,^c^ compared with SIRE 200 mg/kg, and ^d^ compared with SIRE 400 mg/kg.^1^*P* < 0.05,^2^*P* < 0.01, and ^3^*P* < 0.001. SIRE = *Solanum incanum* root extract, DW = distilled water, and GLC = glibenclamide.

**Table 4:** Effect of hydro-methanolic extract of the root of *Solanum incanum* L. in oral glucose-loaded mice.

Group	Blood glucose level (mg/dl)			
	Baseline	30 min	60 min	120 min
DW10	126.35 ± 0.74	185.17 ± 2.10	185.15 ± 2.16^c1d3^	182.53 ± 1.58^c2d3^
SIRE100	127.26 ± 1.24	183.00 ± 1.90	178.21 ± 2.40^d3^	177.13 ± 1.53^d3^
SIRE200	127.28 ± 1.05	184.78 ± 1.46	176.34 ± 1.84^a1^	174.77 ± 1.36^a2d2^
SIRE 400	126.13 ± 1.31	185.83 ± 0.82	172.14 ± 0.80^a3^	165.14 ± 1.39^a3b3c2^
GLC5	127.08 ± 0.80	183.72 ± 1.17	147.62 ± 1.50^a3b3c3d2^	144.65 ± 1.32^a3b3c2d1^

Results are expressed as mean ± SEM (*n* = 6) and analyzed by one-way ANOVA followed by Tukey's post hoc test. ^a^ Compared with negative control, ^b^ compared with SIRE 100 mg/kg, ^c^ compared with SIRE 200 mg/kg, and ^d^ compared with SIRE 400 mg/kg. ^1^*P* < 0.05, ^2^*P* < 0.01, and ^3^*P* < 0.001. SIRE = *Solanum incanum* root extract, DW = distilled water, and GLC = glibenclamide.

**Table 5:** Antihyperglycemic activity of repeated daily doses of *Solanum incanum* L. root hydro-methanolic extract in STZ-induced diabetic mice.

Group	Baseline	Fasting blood glucose level (mg/dl)		Percentage (%) reduction	
		7^th^ day	14^th^ day	7^th^ day	14^th^ day
DC	293.17 ± 1.76^n3^	295.50 ± 0.86^n3^	292.18 ± 1.25^n3^	−0.8%	0.3%
SIRE100	291.00 ± 0.98^n3^	281.85 ± 0.80^n3^	273.55 ± 1.20^a1n3^	3.1%	6.0%
SIRE200	289.12 ± 1.18^n3^	266.82 ± 1.88^a2n3^	253.13 ± 1.10^a2n3^	7.7%	12.4%
SIRE 400	290.17 ± 2.80^n3^	251.42 ± 1.20^a3n3^	233.06 ± 1.37^a3n3^	13.3%	19.7%
GLC5	287.12 ± 2.02^n3^	201.06 ± 1.34^a3n3^	190.32 ± 1.93^a3n3^	30.0%	33.7%
NC	123.09 ± 1.74^a3^	121.51 ± 1.92^a3^	124.23 ± 1.41^a3^	1.3%	−0.9%

Results are expressed as mean ± SEM (*n* = 6) and analyzed by one-way ANOVA followed by Tukey's post hoc test. ^a^ Compared with negative control, and ^n^ compared with normal control. ^1^*P* < 0.05, ^2^*P* < 0.01, and ^3^*P* < 0.001. SIRE = *Solanum incanum* root extract, DC = diabetic control, NC = normal control, and GLC = glibenclamide.

**Table 6:** Effect of hydro-methanolic extract of the root of *Solanum incanum* L. on the body weight of STZ-induced diabetic mice.

Group	Body weight (g)			
	Before induction of DM	Baseline	7^th^ day of treatment	14^th^ day of treatment
DC	31.11 ± 0.80	27.34 ± 0.93^n2^	26.66 ± 1.03^n3^	25.69 ± 1.10^n3^
SIRE100	30.94 ± 0.85	26.78 ± 0.91^n2^	27.79 ± 0.78^n2^	27.91 ± 0.56^n2^
SIRE200	30.84 ± 1.21	27.43 ± 1.11^n2^	28.22 ± 0.72^n2^	31.27 ± 0.53^a1^
SIRE 400	33.14 ± 0.83	28.14 ± 0.44^n2^	31.62 ± 0.65^a2^	32.59 ± 1.41^a2^
GLC5	33.83 ± 0.63	28.45 ± 1.04^n2^	32.34 ± 0.97^a3^	33.23 ± 1.11^a3^
NC	31.13 ± 0.58	32.21 ± 0.79^a2^	33.50 ± 1.15^a3^	34.37 ± 1.35^a3^

Results are expressed as mean ± SEM (*n* = 6) and analyzed by one-way ANOVA followed by Tukey's post hoc test. ^a^ Compared with the diabetic control, and ^n^ compared with the normal control. ^1^*P* < 0.05, ^2^*P* < 0.01, and ^3^*P* < 0.001. SIRE = *Solanum incanum* root extract, DC = diabetic control, NC = normal control, and GLC = glibenclamide.

**Table 7:** Effect of hydro-methanolic extract of the root of *Solanum incanum L*. on serum lipid levels of diabetic mice.

Group	Serum lipid level (mg/dl)				
	STC	STG	LDL-c	VLDL-c	HDL-c
DC	184.74 ± 1.51^n3^	164.32 ± 1.69^n3^	116.99 ± 1.14^n3^	36.59 ± 1.52^n3^	32.90 ± 0.88^n3^
SIRE100	183.16 ± 2.15^n3^	162.12 ± 2.18^n3^	114.20 ± 2.19^n3^	35.03 ± 2.49^n3^	34.11 ± 1.65^n3^
SIRE200	176.10 ± 1.18^a1n3^	154.64 ± 1.46^a2n3^	110.05 ± 0.79^a1n3^	32.14 ± 1.27^n3^	36.14 ± 1.55^n3^
SIRE 400	174.07 ± 0.71^a2n3^	152.92 ± 0.69^a3n3^	107.79 ± 1.01^a2n3^	30.29 ± 1.25^n3^	39.42 ± 0.87^a1n3^
GLC5	172.17 ± 1.12^a3n3^	149.26 ± 1.00^a3n3^	104.27 ± 1.57^a3n3^	27.13 ± 1.52^a2n3^	43.48 ± 1.33^a3n3^
NC	100.93 ± 3.01^a3^	99.92 ± 2.34^a3^	57.58 ± 1.86^a3^	12.06 ± 0.79^a3^	57.02 ± 2.26^a3^

Results are expressed as mean ± SEM (*n* = 6) and analyzed by one-way ANOVA followed by Tukey's post hoc test. ^a^ Compared with the diabetic control, and ^n^ compared with the normal control. ^1^*P* < 0.05, ^2^*P* < 0.01, and ^3^*P* < 0.001. SIRE = *Solanum incanum* root extract, DC = diabetic control, NC = normal control, GLC = glibenclamide, STC = serum total cholesterol, STG = serum triglyceride, HDL-c = high-density lipoprotein cholesterol, VLDL-c = very-low-density lipoprotein cholesterol, and LDL-c = low-density lipoprotein cholesterol.

## Data Availability

The data sets used in this study are available upon reasonable request from the corresponding author.

## Abbreviations

BGL: Blood glucose level
DM: Diabetes mellitus
GLC: Glibenclamide
HDL: High-density lipoprotein
LDL: Low-density lipoprotein
LD_50_: Median lethal dose
OECD: Organization for Economic Cooperation and Development
OGTT: Oral glucose tolerance test
SIRE: *Solanum incanum* root extract
STZ: Streptozotocin
TC: Total cholesterol
TG: Triglycerides
VLDL: Very-low-density lipoprotein
WHO: World Health Organization.
